The article "Ultrasonography Combined with Blood Biochemistry on the Early Diagnosis of Diabetic Kidney Disease" was published in 2022. Journal: Dis Markers.

# Ultrasonography Combined with Blood Biochemistry on the Early Diagnosis of Diabetic Kidney Disease

**DOI:** 10.1155/2022/4231535

**Published:** 2022-10-05

**Authors:** Jing Lin, Guangde Liu, Yuxuan Lin, Chao Wei, Sujun Liu, Youhua Xu

**Affiliations:** ^1^Department of Ultrasound, Guangdong Provincial Hospital of Chinese Medicine-Zhuhai Hospital, Zhuhai, Guangdong, China; ^2^Department of Nephrology, Guangdong Provincial Hospital of Chinese Medicine-Zhuhai Hospital, Zhuhai, Guangdong, China; ^3^Faculty of Chinese Medicine, State Key Laboratory of Quality Research in Chinese Medicine, Macau University of Science and Technology, Taipa, Macao, China; ^4^Macau University of Science and Technology Zhuhai MUST Science and Technology Research Institute, Hengqin, Zhuhai, China; ^5^Zhuhai Hospital of Integrated Traditional Chinese and Western Medicine, Affiliated Hospital of Faculty of Chinese Medicine of Macau University of Science and Technology, Zhuhai, China

## Abstract

**Objective:**

Diabetic kidney disease (DKD) has been well recognized as a microvascular complication of diabetes mellitus. Perfusion of intrarenal arteries is closely related with development of DKD. The aim of the present study was to investigate relation of ultrasonography performance of intrarenal arteries and grade of DKD.

**Methods:**

From May to December at 2021, a total of 54 DKD patients and 36 non-DKD cases were recruited. Ultrasonography performance of intrarenal and arteries at lower extremity was examined by high-resolution ultrasound diagnostic equipment; maximum (Vsmax) as well as minimum (Vdmin) blood velocity of arteries were recorded, and resistance index (RI) of arteries were calculated. Blood routine and biochemical parameters were determined from clinical laboratory of our hospital.

**Results:**

According to eGFR grading, 42.50% of the 54 DKD cases are at Grade 1, and 18.52%, 11.11%, 9.26%, and 18.52% cases were at Grade 2, 3a, 3b, and 4-5, respectively. Blood urea and creatinine were significantly positively related with progress of DKD, while level of Hb was negatively related with DKD. By ultrasonography; we found that Vsmax and Vdmin of main renal artery (MRA), segmental renal artery (SRA), and interlobular renal artery (IRA) were significantly reduced compared with healthy cases; IR of the above arteries was dramatically elevated, and changes of the above data were more obvious than that of lower extremity. Vdmin of MRA, SRA, and IRA was negatively related with grading of DKD, while RI was positively related with the grading. Converging from RI and level of Hb, we found that the level of Hb is positively related with healthy status of the kidney, while RI of the arteries is negatively with that.

**Conclusions:**

Resistance index (RI) of intrarenal arteries, obtained from ultrasonography combining with level of hemoglobin (Hb), is the predictor of progress of DKD.

## 1. Introduction

With the world population aging progress, diabetic kidney disease (DKD) has become a leading contributor to end stage of renal failure (ESRF) [1]. It is estimated that over 30% of patients with diabetes will develop into DKD within 20 years since diagnosis of diabetes [2]. Unfortunately, there is still no way to satisfactory inhibit progress of DKD to now.

Clinically, DKD is arbitrarily diagnosed with appearance and content of proteinuria. For instance, once the urine protein exceeds 300 mg/L or microalbuminuria above 30-300 mg/day, the patients will be clinically diagnosed [3, 4]. However, evidences from two decades have indicated that these two parameters are not specific for DKD [5], and usefulness of proteinuria is facing challenge recently as it lacks sensitivity and specificity in respect of early diagnosis of DKD. On the other hand, DKD has been demonstrated to be positively related with dysfunction of multiple organ systems [6], and most importantly, it will increase cardiovascular events [7]. Currently, definite diagnosis of DKD still relies on renal biopsy and morphological findings. However, severe complication is very common during the invasive operation of renal biopsy, and most cases denied to this operation. Therefore, it is of great significance to develop a method to serve for prediction or early diagnosis of DKD.

DKD has been well recognized as a microvascular complication of diabetes mellitus. Lesion of the vascular wall and decrease of tissue perfusion is the central event during development of vascular disease as well as DKD, and they are positively related with development of DKD. Therefore, seeking a technique that reflects their early changes in cases with diabetes might help early diagnosis of DKD. In the present study, we compiled vascular perfusion of kidney and function of peripheral arteries using ultrasonic diagnosis, and further investigated relationship between grade of DKD and ultrasonic performances. Our current study may supply an noninvasive method and strategy for early diagnosis of DKD in diabetes cases.

## 2. Subjects and Methods

### 2.1. Study Population

All study population were recruited from Department of Nephrology of our hospital from May to December 2021. In general, all newly in-hospitalized DKD cases during the above period that met with the following criteria were included, and all recruited volunteers with non-DKD during this period were included. Finally, a total of 54 DKD patients (23 female and 31 male) aging from 28 to 84 years old (age = 57.72 ± 12.29) and 36 non-DKD cases (23 female and 13 male) aging from 21 to 72 years old (age = 46.78 ± 11.69) were included. All included cases have signed informed consent before study. All study plan, data collection, and ultrasonic operation were approved by Ethics Committee of Guangdong Provincial Hospital of Traditional Chinese Medicine (Approval no. BE2021-122-01).

The inclusion criteria for DKD were as follows: (1) age ≥ 18 years old; (2) DKD was diagnosed according to clinical practice guideline of Kidney Disease Outcome Quality Initiatives (K/DOQI) [8], and (3) no anatomy anomalies in the kidney or peripheral arteries and no renal tumors or renal transplantation.

The exclusion criteria were as follows: (1) malignant tumor; (2) anatomical abnormalities of urinary system; (3) accompanied with urinary or systemic infection.

### 2.2. Laboratory Data

All laboratory data were obtained from clinical laboratory of Guangdong Provincial Hospital of Chinese Medicine-Zhuhai Hospital. Estimated glomerular filtration rate (eGFR) was determined according to the following equation: eGFR = 186 × Scr^−1.154^ × (age)^−0.203^ [×0.742 (if female)]. Staging of DKD is as follows: (1) Grade 1: eGFR ≥ 90; (2) Grade 2: 89 ≥ eGFR ≥ 60; (3) Grade 3a: 59 ≥ eGFR ≥ 45; (4) Grade 3b: 44 ≥ eGFR ≥ 30; (5) Grade 4: 29 ≥ eGFR ≥ 15; (6) Grade 5: eGFR < 15.

### 2.3. Ultrasonic Investigation of the Participants

Real-time ultrasonography at B-mode was carried out in each participant using a high-resolution ultrasound diagnostic equipment (Phillips) by well-trained and validated examiners. Maximum (Vsmax) as well as minimum (Vdmin) blood velocity of arteries of lower extremity including common femoral artery (CFA), superficial femoral artery (SFA), popliteal artery (POA), anterior tibial artery (ATA), posterior tibial artery (PTA), peroneal artery (PEA), dorsalis pedis artery (DPA), arteries within the kidney including main renal artery (MRA), segmental renal artery (SRA), and interlobular renal artery (IRA), at both sides were recorded. Resistance index (RI) of the arteries was obtained according to the following equation: RI = (Vsmax − Vdmin)/Vsmax. Mean value of the right and left side of the above values were obtained for further analysis.

### 2.4. Statistical Analysis

Data are expressed as mean ± SD or otherwise indicated. Data are analyzed by GraphPad Prism 9 using *t*-test or one-way ANOVA. Multiple linear regression of the data was obtained by GraphPad Prism 9. *P* values <0.05 is considered to be statistically significant.

## 3. Results

### 3.1. Overview of the Participants

A total of 36 healthy as well as 54 DKD cases were included in this study. Within the DKD cases, 42.59% were female, and 62.96% were between 41 and 65 years old (Table 1). According to eGFR grading, 42.50% of the DKD cases are at Grade 1, and 18.52%, 11.11%, 9.26%, and 18.52% cases were at Grade 2, 3a, 3b, and 4-5, respectively (Table 2). As shown in Table 2, once the cases progress into grade 3, levels of blood urea and cr were significantly increased, while Hb was decreased.

### 3.2. Blood Velocity and Artery Resistance Index Was Altered in DKD Cases

To firstly evaluate haemorheological changes of renal arteries for DKD cases, maximum (Vsmax) as well as minimum (Vdmin) blood velocity of main renal artery (MRA), segmental renal artery (SRA), and interlobular renal artery (IRA) were recorded. As shown in Figure 1, the maximum and minimum blood velocity of MRA, SRA, and IRA was significantly decreased in DKD cases compared with healthy control; moreover, resistance index (IR) of the above arteries was dramatically elevated (*P* < 0.001 vs. ctl). These data suggested that renal perfusion was reduced in DKD.

To further determine changes of arteries in lower extremity, Vsmax in common femoral artery (CFA), superficial femoral artery (SFA), popliteal artery (POA), anterior tibial artery (ATA), posterior tibial artery (PTA), peroneal artery (PEA), and dorsalis pedis artery (DPA) was analyzed. As shown in Figure 2, Vsmax in CFA and SFA was significantly reduced in DKD cases (*P* < 0.05 vs. ctl), but no statistical significance was found for Vsmax in other arteries at lower extremity.

Converging with the above data, ultrasonic changes of CFA as well as arteries within the kidney were related with DKD to some extent.

### 3.3. Ultrasonographic Changes of CFA and Arteries within the Kidney of DKD Cases

To explore relation of ultrasonographic changes of CFA and arteries within the kidney of with grading of DKD, Vsmax, Vadmin as well as RI of the arteries were analyzed. As shown in Figure 3, Vdmin of MRA, SRA and IRA was negatively related with grading of DKD; while RI was positively related with the grading. More importantly, a more significance was found once the grading progressed into ^″^3^″^. No statistical significance was found in Vsmax or ultrasonographic changes of CFA concerning their relation with DKD grading.

### 3.4. Multiple Regression Analysis of the Data

Converging from the above data, we can conclude that Hb and RI are two pivotal parameters that closely related with grading of DKD. To further define correlation among the data above, multiple linear regression analysis was conducted. As shown in Figure 4, level of Hb is positively related with healthy status of the kidney, while RI of the arteries is negatively with that.

## 4. Discussion

With the aging progression around the world, diabetic kidney disease (DKD) has becoming one of the major reason that contributes to end stage renal disease (ESRD). Although it has been well recognized that early-diagnosis is pivotal to inhibit progression of DKD, a noninvasive, real-time, and dynamic method that reflect status of the kidney is still rare. In the present study, we supplied an equation that reflect correlation among eGFR, resistance index of arteries within the kidney, and level of Hb. Our present finding may help clinicians for early diagnosis and treatment of DKD.

It was reported that about 30-40% of cases with type 2 diabetes mellitus are likely to have kidney lesion [9]; more importantly, this lesion is believed to be irreversible [10]. In this sense, early diagnosis is pivotal. Currently, biopsy is still the gold standard for diagnosis of DKD and most other renal diseases [11]. However, most of the cases are not evaluated by biopsy due to its invasive test and possible severe side effects [12], and clinical symptoms converging with laboratory data are applied for diagnosis. In the current study, all DKD cases are clinically diagnosed, and stage of the disease was obtained according to the eGFR value.

It has been well recognized that decreased perfusion of the kidney plays a key role in the development of DKD [13]. A finding from Ma et al. indicated that the perfusion velocity of the microcapillary bed within the kidney in DKD cases is significantly reduced [14]. Ultrasonography is a noninvasive method that has been widely applied to evaluate morphology changes as well as hemorheology of the organism. We found that both maximum and minimum blood velocity of arteries within the kidney were significantly reduced with grading of DKD, while the resistance index of intrarenal arteries was increased. Although blood velocity in arteries of lower extremity is also altered, there is no statistical significance among different grades of DKD.

It has been well understood that hemoglobin (Hb) production is closely related with secretion of erythropoietin (EPO). Recent findings have found reduced EPO, and anemia are independent risk factors for microvascular diseases including DKD [15–17]. In the present study, we found that Hb is negatively related with grading of DKD; this is in line with previous findings. Compelling with resistance index (IR) of intrarenal arteries, we further obtained a regression equation, and found that the level of Hb is positively related with eGFR, while RI of intrarenal arteries is negatively with that.

It should be noted that as there is still no well recognized ultrasonography that predict progress of the damage of kidney; the current finding is just an alternative for clinicians, and it cannot replace the gold standard of biopsy on diagnosis of renal damage. On the other hand, recent advances in finding biomarkers of early DKD in diabetic population by omics and molecular-biology also supplied an alternative method. For instance, long noncoding RNAs (lncRNAs) have been suggested to play a role in early development of DKD [18], and glycated peptides within the urine may predict dysfunction of proximal tubule within the kidney [19].

In summary, we show in the present that resistance index (IR) of intrarenal arteries obtained from ultrasonography combining with level of hemoglobin (Hb) are predictor of grading DKD. Our present finding supplied an alternative and noninvasive method for early diagnosis of DKD.

## Figures and Tables

**Figure 1:** Ultrasonography characteristic of renal arteries in DKD cases. Main renal artery (MRA), segmental renal artery (SRA), interlobular renal artery (IRA). ∗p<0.05, ∗∗∗p<0.001, ∗∗∗∗p<0.0001.

**Figure 2:** Ultrasonography characteristic of arteries in lower extremity of DKD cases. Common femoral artery (CFA), superficial femoral artery (SFA), popliteal artery (POA), anterior tibial artery (ATA), posterior tibial artery (PTA), peroneal artery (PEA), dorsalis pedis artery (DPA). ∗p<0.05, ∗∗∗∗p<0.0001.

**Figure 3:** Ultrasonographic changes of arteries within the kidney are related with grading of DKD. Main renal artery (MRA), segmental renal artery (SRA), interlobular renal artery (IRA). ∗p<0.05, ∗∗p<0.01, ∗∗∗∗p<0.0001.

**Figure 4:** Multiple regression analysis of the eGFR against RI and Hb.

**Table 1:** Characteristics of the subjects.

	Control (*n* = 36)	DKD (*n* = 54)	*P* values
Mean age (SD), *y*	47.42 ± 12.15	57.72 ± 12.29	<0.001
Age, *n* (%)			<0.001
≤40 y	10 (27.78)	5 (9.26)	
41-65 y	20 (55.56)	34 (62.96)	
>65 y	1 (2.78)	16 (29.63)	
66-70 y	0	8 (14.81)	
71-75 y	1 (2.78)	5 (9.26)	
76-80 y	0	2 (3.70)	
>80 y	0	1 (1.85)	
Women, *n* (%)	23 (63.89)	23 (42.59)	0.0054

**Table 2:** Laboratory characteristic of DKD participants (mean ± SD).

	Grade 1	Grade 2	Grade 3a	Grade 3b	Grade 4-5	*P* values
*N* (%)	23 (42.59)	10 (18.52)	6 (11.11)	5 (9.26)	10 (18.52)	
Hb	139.74 ± 17.59	131.00 ± 23.31	127.83 ± 15.82	101.20 ± 8.84	93.90 ± 9.96	<0.001
FBG	8.51 ± 2.96	7.90 ± 1.77	9.88 ± 6.90	8.37 ± 1.59	7.31 ± 3.30	0.7881
HbA1c (%)	7.87 ± 2.42	8.97 ± 3.98	8.50 ± 3.88	8.06 ± 2.80	6.49 ± 0.84	0.4250
Blood urea (mmol/L)	4.96 ± 1.54	6.35 ± 2.70	6.46 ± 1.91	13.45 ± 3.89	19.96 ± 7.41	<0.001
Blood Cr (*μ*moI/L)	68.28 ± 21.05	85.28 ± 14.03	111.67 ± 20.12	154.62 ± 18.96	520.11 ± 247.32	<0.001
eGFR	113.12 ± 18.99	77.63 ± 9.20	52.71 ± 4.08	38.20 ± 3.91	11.58 ± 6.81	<0.001

Note: eGFR = 186 × Scr^−1.154^ × (age)^−0.203^ [×0.742 (if female)]. FBG: fasting blood glucose; Cr: creatinine; eGFR: estimated glomerular filtration rate.

## Data Availability

The original data can be obtained from the corresponding author upon reasonable request.
